# Performance Optimization of Industrial Supply Chain Using Artificial Intelligence

**DOI:** 10.1155/2022/9306265

**Published:** 2022-07-30

**Authors:** Madani Abdu Alomar

**Affiliations:** Department of Industrial Engineering, Faculty of Engineering-Rabigh, King Abdulaziz University, Jeddah 21589, Saudi Arabia

## Abstract

Nowadays, organized retailing has witnessed a newer trend in the upcoming generations. Globally, these changes are attributed to growing family income, increased female participation, the transformation from joint to nuclear family structure, and technological advancements. Moreover, other variables such as lower supply chain costs, growing sales, rising consumer demands, changing market structure, and increasing competition also influenced supply chain networks. It is observed that the organizational nonlivestock supply chain performance is affected by strategic, operational, and environmental aspects. AI is helping to deliver powerful optimization capabilities, which are required for more accurate capacity planning, improved productivity, high quality, lower costs, and greater output, all while fostering safer working conditions. These benefits are all made possible thanks to the introduction of AI in supply chains. By conducting a comprehensive analysis of the relevant previous research, the purpose of this work is to determine the specific contributions that artificial intelligence (AI) has made to supply chain management. This research attempted to discover the present as well as possible AI strategies that may increase both the study of Supply Chain Management as well as the practice of it. This was done in order to solve the current scientific gap of AI in Supply Chain Management. It was also found that there are holes in the existing study that need to be filled by more scientific investigation. To be more exact, the following four facets were discussed: (1) the AI approaches that are most often used in Supply Chain Management; (2) the AI techniques that have the potential to be used in Supply Chain Management; (3) the Supply Chain Management subfields that have benefited from the application of AI so far; and (4) the subfields that have a high potential to be improved by AI. Identifying and evaluating articles from the four supply chain management domains of logistics, marketing, supply chain management, and manufacturing require the use of a predetermined set of inclusion and exclusion criteria. In this study, insights are provided via the use of methodical analysis and synthesis. A better understanding of these parameters not only improves the nonlivestock supply chain processes but also ensures competitive advantage. The present research aims to test the following elements that including supply chain speed, customer retention, supply chain management integration, and various management. The proposed work categorizes the performance of the supply chain using the Improved Feed Forward Network with Particle Swarm Optimization technique. Results indicate that inventory management, customer happiness, profitability, and client base identification are listed as competitive advantage elements. On the other hand, stakeholder satisfaction, innovation and learning, market performance, customer satisfaction, and financial success are the six recognized organizational performance criteria. Resultantly, the overall performance metrics of the proposed work is 94.12%, while accuracy rate, specificity, and sensitivity rate are found to be 94.12%, 92.15%, and 89.14%, respectively. The research can be helpful for industrial managers to optimize the performance of supply chain systems using artificial intelligence.

## 1. Introduction

A supply chain is comprised of all of the actions that go into satisfying the needs and requests of customers. From the stage of raw materials to the stage of finished products, these activities are related to the movement and transformation of commodities, information, and finance flows. “A supply chain is a network of facilities and distribution options that performs the functions of procurement of materials, the transformation of these materials into intermediate and finished products, and the distribution of these finished products to customers.” “A supply chain is a network of facilities and distribution options that performs the functions of transformation of these materials into intermediate and finished products” [1].

Even though the effect that manufacturing activities have on the natural environment is a major cause for concern in developed nations, very little is known about the consequences of manufacturing activities in developing nations. This is despite the fact that industrial operations have a significant impact on natural environments. The industrial sector in developing countries is especially polluting, which has led to a large rise in the amount of pressure that is being imposed on the environment. The deterioration of the environment and increased pressure suggest that stringent environmental rules should be implemented in emerging nations in order to prevent environmental degradation from occurring simultaneously with economic growth [2]. Such rules would prevent environmental degradation from occurring simultaneously with economic growth. Only through the conscientious management of natural resources and the implementation of environmentally responsible practices can this goal be attainable. The discharge of ecologically hazardous goods and contaminated gases into the environment may be traced back to the industrial sector. According to the Environmental Protection Agency (EPA), in order for manufacturing companies to lessen their impact on the environment caused by polluting gases and hazardous products, they must integrate a “green component” into their production processes and management systems for supply chains (SCM). In order to protect the environment from being harmed, stricter environmental regulations need to be implemented as soon as possible. As a consequence of this, new paradigms in SCM were developed, and now they are known as green supply chain management (GSCM). The term “green supply chain management” (GSCM) may be described as the practice of introducing environmentally aware thinking into “supply chain management.” The process begins with the creation of environmentally friendly products and continues on via strategic sourcing, procurement, environmentally friendly manufacturing practices, and eventually the delivery of finished goods and services to customers. It also includes the management of materials after they have outlived their usefulness and the reuse of those materials [3]. In the field of global supply chain management, there has been an increased emphasis on environmentally responsible purchasing since the 1990 s (GSCM). Reference [4] looked into how the goods they made impacted the surrounding environment and reported their findings. The concept of “green purchasing,” which promotes the purchase of raw materials that are less harmful to the environment, was conceptualized as a result of this study. When it comes to the acquisition of raw materials (point 5), environmental factors are taken into account, with a special focus placed on the recycling of finished goods. The governing body of the Chartered Institute of Purchasing and Supply (CIPS) and Business in the Environment was established in 1995 with the primary objective of assisting organizations in striking a balance between commercial activities and environmental impact by increasing the efficiency of supply chain management. This goal was originally established with the intention of assisting organizations in striking a balance between commercial activities and environmental impact.

According to the United Nations Development Programme [5], if every citizen of the world lived a life that was comparable to the standard of living enjoyed by citizens of an industrially developed country, which is not equivalent to the 20% of the current population, the global population would consume nearly three to six planets every year. This is not equivalent to the 20% of the population that currently lives that kind of life. Reference [6] estimates that by the end of the year 2025, the population of the Earth will have expanded to 8.3 billion people from its current count of 7.6 billion. There is a rising demand for natural resources (such as materials and energy) as a result of the expanding population, which leads to a fast depletion of natural resources and the formation of dangerous living situations around the globe. This fast loss of natural resources will further contribute to the destruction of the environment, which will include, among other things, contaminated gases, air, water, and soil. The industrial manufacturing sector not only makes a major contribution to the expansion of the country's economy, but it also has an immediate bearing on the quality of life enjoyed by the country's citizens as well as the Gross Domestic Product (GDP) of the country (GDP). The manufacturing sector is the most important sector in every country because it is the sector that is responsible for meeting the most fundamental needs of humanity. It is also the sector that contributes the most to sustainable development because it is the sector that provides the necessary goods and services. In order to create output, the manufacturing sector has to begin with input. In this input–output system, the input is raw material in the form of natural resources, and the output is the result of the transformation that the raw material is used to create. These natural resources are converted into finished or semifinished products by using a wide variety of firms that are involved in the manufacturing process [7]. Energy and raw materials are the two most essential components that a manufacturer might have available to them. The production of energy and goods, which are subsequently recycled, requires the use of natural resources such as fossil fuels and ores, among other natural resources. Every country, whether it is considered to be developing or already developed, is making every effort to increase the quality of life of its citizens and the families they support. At the same time, technologically sophisticated governments do not make any sacrifices to the high standard of living that these nations have already created [8]. As a result, the graph that follows demonstrates that the average rate of resource depletion on a worldwide scale is growing at the same time as the living standards of people all over the world are improving. As a direct consequence of this, there is a significant and unavoidably high level of demand for products that are produced in the manufacturing sector. Unluckily, this unavoidable situation is already on its way to becoming into a major challenge that is difficult to control. Reference [9] estimates that the manufacturing industries are responsible for approximately half of all global energy consumption and that the depletion of natural resources (such as metals like iron and wood, lead, aluminum, nickel, copper, and others) used by these manufacturing industries is increasing at an alarming rate on a global scale. Reference [9] also estimates that the energy consumption of the manufacturing industries accounts for approximately half of all global greenhouse gas emissions. The amount of money that people spend on products and services is growing at a pace that is comparable to an exponential curve. As a direct consequence of this, the industrial sector has been increasing at an exceptionally quick pace. After launching the most ambitious programme in the country's history, “Make in India,” to enhance the country's economy, a developing nation like India, in particular, is making every effort to achieve rapid industrial development. This is especially the case after launching the “Make in India” initiative. The rise of the industrial sector will lead to an increased demand for natural resources, which in turn will lead to an increase in environmental pressures. These pressures will continue to build as long as the demand for natural resources remains high. This is the most significant challenge that every country on Earth is now facing. In order to forestall anything like this from occurring, nations all over the globe need to develop rules and regulations that are very strict. As a consequence of this, the industrial sector, the academic world, government agencies, and international community's all face a significant challenge when attempting to lessen the risks to the environment while simultaneously fostering economic expansion [10]. The corporations are up against a challenging task in order to achieve a more rapid growth in the Indian manufacturing sector without negatively impacting the environment. It is possible for India to achieve a level of ecological advancement on par with that of other industrialized countries if manufacturing companies in the country adopt the concepts of GSCM. In spite of the fact that putting these GSCM ideas into practice is not always easy, especially in countries that are poor and underdeveloped, it is essential to have an understanding of the factors that drive Indian manufacturing to adopt GSCM approaches. In addition to this, it is of the utmost importance to recognize and comprehend the factors that produce obstacles in the process of GSCM procedure adoption. The aforementioned problems are what people mean when they talk about “barriers to GSCM deployment” [11]. It is very necessary to take measures to lessen the influence of any potential roadblocks in order to make certain that the GSCM principles are effectively adopted. It is equally necessary to look at the processes and practices that assist to lower-environmental risks in the supply chain throughout the research process, even when the primary focus of the study is on the drivers and the impediments. In common parlance, these activities are known as GSCM practices [Citation needed]. Because of this research, manufacturing companies in India will be able to incorporate environmental considerations into their supply chains, which suggest that manufacturing operations can be carried out while keeping the environment, the economy, and the society in mind [12], as shown in the study. This research will be beneficial to these companies. Given the aforementioned information, the purpose of the ongoing research project is to explore the drivers, barriers, and green practices of GSCM in the context of the Indian manufacturing sector. In order to acquire information on the drivers, difficulties, and practices of global supply chain management (GSCM) in Indian manufacturing enterprises, a questionnaire survey would be employed.

## 2. Literature Review

According to Chirstmann and Taylor's (2001) results in their research, export and commerce with foreign clients are the most important drivers of improvement in environmental conditions in Chinese industry. This is according to the findings of Chirstmann and Taylor's study. Reference [13] came to the conclusion that the adaptation and expansion of a “Environment Managerial System” (EMS), as well as the accomplishment of a favorable outcome, are mostly reliant on the management direction of the company and its level of environmental awareness. In a manner comparable to this, top management is accountable for being aware of environmental concerns and ensuring that these concerns are resolved in the industries in which they are employed. These standards, which were uncovered over the course of the investigation, are relevant to each and every sector. According to the findings of their research, the European Union (EU) has mandated that any new “Electricals and Electronics Equipment” (EEE) that is brought onto the market cannot contain any of six toxic compounds. These compounds are lead, cadmium, mercury, hexavalent chromium, polybrominated diphenyl ether, or polybrominated biphenyls. According to [14], businesses will not be able to continue operating unless they remove actions and materials that are damaging to the environment from their production processes. As a consequence of their research, [15] found that industrial businesses have started to recognize the advantages that come with adopting a more realistic perspective when it comes to environmental policy. These manufacturing organizations can only be turned into environmentally aware businesses if they are able to improve their corporate image while simultaneously reaping the advantages of resource efficiency. Additionally, it has been observed that the quality of human resources, support from the corporation, pressure from regulatory organizations, and aid from the government are all factors that contribute to the adoption of environmentally friendly activities. In a manner comparable to this, it is possible to demonstrate, based on the assessment of the relevant literature, that these features have a very stimulating impact on the efficient adaptation of environmentally friendly operations in the Chinese logistics industry. He observed in his analysis that the size of a company, the authority of the shareholders of that company, and environmental regulations are all associated with environmental problems. These problems have been uncovered on several occasions by researchers in the course of their studies. Reference [16] found a new important business difficulty that has recently arisen across a variety of businesses; they refer to this problem as the “new big business challenge.” The integration of environmental, social, and economic viewpoints into supply chain management is widely considered to be an essential step for enterprises to take toward achieving sustainable development. This viewpoint has widespread support from a wide range of stakeholders. According to the findings of an investigation, [18] found that the pressure exerted by the market is the single most significant driver of the adoption of GSCM procedures in the Chinese automobile manufacturing sector. According to their findings, “employee motivation, health and safety” is the most significant driver in the production of two-wheelers, whereas “government regulations and laws” is the most significant driver in the production of four-wheelers. Both of these factors are important in the manufacturing of four-wheelers. Environmental, global climate, and consumer awareness were all considered to be of equal importance when it came to the implementation of GSCM processes in general industrial sectors. According to Huang et al. [18], customer demand, pressure, and awareness from suppliers, as well as rules passed by the Chinese government, are all factors that are driving Chinese SMEs to embrace concepts of global supply chain management. According to the study, it was also shown that different sectors have a variety of different motivations for the use of GSCM approaches. The key reasons are the development of new technology, the enforcement of existing regulations, the cultivation of a green image, the dedication of management, and the introduction of new laws. They came to the conclusion that industry-specific research should get a greater amount of focus, and that this should be done so that the sectors that are the most harmful to the environment may be addressed first. This is particularly true in emerging nations since the economies of these countries are still in the formative phases of growth. According to [19], the introduction of GSCM in leather enterprises in northern Tamil Nadu is being pushed by both crucial and obtrusive aspects. This was discovered by the researchers. Structural equation modeling is the foundation of the model that is built using Vikor and Fuzzy VIKOR as its building blocks (SEM). These things need to be taken into account in order for GSCM activities at any level to be carried out in an efficient manner. Nonmembers, organizational members, upward stream members, and downward stream members are the four aspects of the supply chain that should be considered. Reference [20] found that there are 14 drivers of GSCM that have a substantial influence on the execution of the GSCM 26 recommended practices by conducting a study of the relevant literature. As a result of the findings of this analysis of the relevant literature, it would seem that regulations, the demand of consumers, and competition are the most important drivers of global supply chain management.

An attempt has been undertaken to conduct a study of the literature on various performance indicators for global supply chain management. This study will be based on previous research (GSCM). According to the research that has been done, there are primarily three different types of performance metrics that may be used for GSCM. There are three distinct categories of drivers: drivers, obstacles, and environmentally responsible business practices. The results of the literature review uncovered some holes that need to be filled, which are summarized below. There is no study that has been published in the Indian context that depicts the hierarchy and interaction between the various performance measures of the Global Supply Chain Management (GSCM). GSCM stands for “global supply chain management.” A significant number of the studies that have been published have focused their attention on a limited number of GSCM performance metrics rather than taking into account the wide variety of performance measures that can be broken down into three categories: drivers, barriers, and environmentally friendly practices. At the moment, there is no study that has been published in the relevant literature that assesses various performance measures based on how relevant they are from a variety of perspectives. In the present research, there are four primary points of view that have been taken into account in order to evaluate the various performance criteria. These four perspectives are the most essential participants in the process of implementing GSCM in India's manufacturing industry, which is now in the process of doing so. According to the findings of the investigation of the relevant literature, there are only a small number of studies that can be found in the relevant literature that have produced models for the various performance indicators making use of Exploratory Factor Analysis up to this point. In addition, a confirmatory factor analysis is carried out in order to validate the EFA model that has already been developed. In light of the findings made above, there is a glaring lack of concerted effort being put out to explore the various performance measures of GSCM with the intention of establishing the impact that these metrics have on the industrial sectors. The current research endeavor makes an attempt to investigate the various performance indicators of GSCM and their influence on the manufacturing sectors in order to facilitate the adoption of GSCM in a rising globalized and competitive environment in the context of India. This is done in an effort to make the adoption of GSCM easier in a globalized and competitive environment. The goal of this research was to carry out a questionnaire survey in order to investigate the many performance indicators that are used by manufacturing companies in India. In spite of the fact that a number of studies that are comparable have been reported in the published study, there is an undeniable need for more research that is more in-depth regarding the many performance indicators of GSCM in the context of India.

## 3. Materials and Methods

This research takes into account four phases in the supply chain: vendors, production facilities, warehouses, and distribution centers. These steps are listed in the order of their importance to the supply chain in this study attempt. On benchmark tests, it should be noted that when compared to other algorithms, the Non-Linear Inertia Weight Particle Swarm Optimization (NLIW-PSO) method surpassed other PSO versions as well as the Genetic algorithm with good performance. Prior chapters discussed the details of comparative evaluation for the three-echelon supply chain network problem, which was carried out using all PSO variants and GA. It was shown that the NLIW-PSO outperformed all of the other PSO variations and all of the GA in the previous section. Because of this, a technique known as nonlinear inertia weight particle swarm optimization (NLIW-PSO) has been developed for the aim of optimizing the four-echelon supply chain architecture in this research. When it comes to the supply chain network, the total supply chain operating cost (TSCC) and profit of the supply chain network are considered to be performance indicators.

### 3.1. Dataset

The automotive industry throughout the globe seems to be undergoing unplanned shifts, with the enhancement of supply chains being one of the primary areas of concentration alongside the reduction of costs, the optimization of processes, and the enhancement of timely throughput. Having an efficient traceability system in place is the general success metric that must be reached in order to get a superior output in all of the aforementioned priority areas. In the automobile business, “traceability” refers to a system that documents the lineage of the individual components that went into the production of a certain item. Even if businesses have committed a significant amount of resources toward the goal of improving their supply chain and establishing traceability, it has been observed that these businesses still have little visibility and insight into their supply chain at any particular instant. [Case in point] This study intends to utilize blockchain technology in order to eliminate inefficiencies that are present in conventional automotive supply chains. These inefficiencies can be eliminated by increasing transparency, streamlining processes, and decentralizing the network. Additionally, this study will provide stakeholders and companies with a host of value-adding features that will ensure transactions are completed more quickly and smoothly. The research highlights the benefits that may be gained by enabling automotive supply chains with blockchain technology. The establishment of the aforementioned network is accomplished with the help of Hyperledger Composer.

### 3.2. Methods of Input Tuning Data

There are four components to this objective function (Equations 4.1 to 4.4). It is included in the first part, named overall supplier cost of material (TSMC), that the overall cost of raw materials from all suppliers to the production units are included. Entire total transportation cost (TTC) refers to the total transportation cost incurred from all 139 suppliers to plants, as well as the total transportation cost incurred from plants to warehouses, which is shown in the second portion of the table. In the manufacturing industry, TMC is an abbreviation for Total Manufacturing Cost incurred at the plants, and TWC is an abbreviation for Total Warehouse Cost, which includes the costs of maintaining warehouse inventory as well as the costs of shipping finished goods from warehouses to respective distribution centers in order to meet demand. The total manufacturing cost (TMC) and the total working cost (TWC) are two components of the total manufacturing cost (TMC).

In order to compute the second objective function, which is the total supply chain network Profit (PROF), it is split into five sections (equations 4.1 to 4.4 and equation 4.7) and multiplied together (equation 4.9). To begin, the total revenue generated by sales at warehouse distribution centers is represented by half of the equation. The total supplier material cost will be shown in the second part of the report (TSMC). The total transportation costs (TTC) incurred from all suppliers to plants, as well as the total transportation costs (TTC) incurred from plants to warehouses, are included in the third part. The fourth component represents the total manufacturing cost (TMC) borne by manufacturing facilities. In order to fulfil demand, the fifth component, total warehouse costs (TWC), comprises of the expenses of inventory holding at warehouses as well as the costs of delivering completed items from warehouses to distribution centres. In order to fulfil demand, the total warehouse cost (TWC) is computed as the sum of inventory carrying costs at warehouses and the shipping costs of completed items from warehouses to distribution centres. TWC is calculated as a percentage of the total warehouse cost.

(a) Total supplier materials cost
  (1) $$\begin{array}{c} \text{TSMC}=\sum_{c}\sum_{v}\sum_{p}\left(CS_{c,v}\times X_{c,v_{p}}\right). \end{array}$$
(b) Total transportation cost
  (2) $$\begin{array}{c} \text{TTC}=\sum_{c}\sum_{v}\sum_{p}\left(X_{c,v,p}\times {\text{STC}}_{c,v,p}\right)+\sum_{p}\sum_{w}Y_{p,w}\times {\text{PTC}}_{p,w}. \end{array}$$
(c) Total manufacturing cost
  (3) $$\begin{array}{c} \text{TMC}=\sum_{p}\left\{\left(MC_{p}\right)\times \left(\sum_{w}Y_{p,w}\right)\right\}+\left\{\sum_{p}\left(IC_{p}\times \sum_{c}I_{c,p}\right)\right\}. \end{array}$$
(d) Total warehouse cost
  (4) $$\begin{array}{c} \text{TWC}=\sum_{w}\sum_{d}\left(Z_{w,d}\times {\text{WTC}}_{w,d}\right)+\sum_{w}\left({\text{WIC}}_{w}\times I_{w}\right). \end{array}$$
(e) Total supply chain operating cost
  (5) $$\begin{array}{c} \text{TSCC}=\text{TSMC}+\text{TTC}+\text{TMC}+\text{TWC}. \end{array}$$
(f) Profit of SCN
  (6) $$\begin{array}{c} \text{PROF}=\sum_{d}\left(D_{d}\times SP_{d}\right)=\text{TSCC}. \end{array}$$
(g) Revenue generated by SCN
  (7) $$\begin{array}{c} \text{REV}=\sum_{d}\left(D_{d}\times SP_{d}\right), \end{array}$$
  (8) $$\begin{array}{c} \text{TSCC}=\text{TSMC}+\text{TTC}+\text{TSX}-\text{TWC,} \end{array}$$
  (9) $$\begin{array}{c} Min\text{TSCC}=\left[\sum_{v}\sum_{v}\sum_{\eta }\left({\text{CSS}}_{+\infty }\times X_{\text{car}}\right)\right]+\left[\sum_{z}\left\{\left(MC_{,},x\left(\sum Y_{me}\right)\right)\right\}+\left\{\sum^{n}-\left(x_{,},\sum I_{ce}\right)\right\}\right]+\left[\sum_{\alpha }\sum_{\alpha }\left(Z_{\alpha ,}\times {\text{WTC}}_{\alpha ,\lambda }\right)+\sum_{v}\left(WC_{\alpha }\times I_{\alpha }\right)\right], \end{array}$$
  (10) $$\begin{array}{c} \text{PROF}=\sum_{a}\left(D_{4}=SP_{4}\right)-\sum_{V}X_{\text{one }}\leq L_{\text{loper }}Vc_{v}, \end{array}$$
  (11) $$\begin{array}{c} \sum_{p}Y_{nw}\leq U_{p}vw, \end{array}$$
  (12) $$\begin{array}{c} \sum_{v}Z_{n}\leq V_{v}v_{d}, \end{array}$$
  (13) $$\begin{array}{c} \sum_{v}Z_{x}=D_{d}vd. \end{array}$$

### 3.3. Feed Forward Neural Network

In the proposed algorithm, the network learning parameter is first initialized. Here, the change of weight for output layer and hidden layer is determined using cost function equations (5.7) and (5.8). respectively.

**Step 1 .**

Initialize the parameter to some random values

**Step 2 .**

Assign Threshold value to a fixed value based on the sigmoid function.

**Step 3 .**

Calculate linear output using equation (5.2)

**Step 4 .**

Calculate non-linear output using sigmoid function as in equation (5.3)

**Step 5 .**

Calculate weight change for output layer using equation (5.7)

**Step 6 .**

Calculate the weight change for hidden layer using equation (5.8)

**Step 7 .**

Calculate the mean square error

**Step 8 .**

If the mean square error value is greater than threshold value, then the above steps from 3 to 7 is repeated

**Step 9 .**

If the mean square error value is less than threshold value, then declare that the network is trained

Figure 1 indicates the proposed network architecture applied in this research.

## 4. Results and Discussion

The ideal mathematical model presented in this section was implemented with the help of the MATLAB simulation programme. This model was then used to showcase the optimal A supply chain data approach in PMU, as seen in Figure 2. This method utilises the second-order Kalman filter, often known as the SOKF, to monitor the signal phasor throughout the PMUs that were spread out over the grid. In order to show the robustness of the model that is being considered, the simulation work for the proposed strategy comprises putting the method through its paces in a range of different situations. Because of this method, the amount of phase error that occurs is reduced to an acceptable level. Keep in mind that the following figures are derived from the correlation that exists between phase, measured in radians, and the total number of samples.

The proposed method in the PMU has been considered in the presence of Gaussian noise, as shown above in Figure 2, where the second-order Kalman filter has picked up the value of the supply chain data because it takes a larger number of samples with very close results to the reference phase, where the supply chain data results have performed better and are closer to the reference phase than the Supply chain data, as represented by the blue line in the figure, where the Supply chain data results have performed better than the Supply chain data, as represented by The use of MSE to evaluate the performance of the proposed approach based on SOKF, which was shown to be able to better monitor the phase of the system in the presence of Gaussian noise, demonstrates that the suggested model performs very well in the presence of Gaussian noise. This is shown by the fact that the proposed approach is able to better monitor the phase of the system in the presence of Gaussian noise. Take into consideration the fact that the improvement is 21.45 percent under Gaussian noise when measured at a rate of 5 dB, which is a considerable gain.

On the other hand, when there was non-Gaussian noise present, the outcomes of the simulation were taken into account and shown in Figures 3 and 4. The resilience and effectiveness of the optimum method SOKF, which was developed by the PMU, was demonstrated by the fact that the Supply chain data technique in the PMU has outperformed the Synchrophasor approach under extreme environmental circumstances. This shows that the optimum method SOKF was developed by the PMU. In the presence of non-Gaussian noise, the SOKF approach performed much better than the prior model, as shown by MSE's analysis. This is in comparison to the performance of the current model. Because of this, the presence of SOKF in place of non-Gaussian noise is absolutely necessary in order to get the outcomes that are intended. It is plain to observe that the presence of non-Gaussian noise brings to an increase of 16.2 percentage points in the rate at 5 decibels.

Similarly, the multi objective analysis was performed for the second set of objectives, which were TSCC and GMROI for the four stage multi echelon supply chain network architecture. Assuming that the objectives had different weights but were of equal importance, the performance analysis was carried out for the different service levels, which were 50%, 84%, 97%, and 99.9%, and the results are tabulated in Table 1.

The decision-making elements that are linked with the various service levels are listed in Table 1, and each component has been given the same weightage. As a result of the findings of the multi-objective performance analysis that was presented earlier, it is possible to draw the conclusion that as service levels increase, the TSCC of SCN also increases. On the other hand, as service levels increase, the GMROI decreases. This is due to the fact that all warehouses are required to maintain safety stock, the quantity of which varies depending on the required service level. SCN has a gross margin (GMROI) that ranges from 2.8 to 3.6, and its total sales cost (TSSC) falls somewhere in the range of Rs. 12,37,000 to Rs. 19,78,000, depending on the service level. In order to fulfil his or her needs (service levels to meet consumer demand), the decision maker may make a choice that is understandable based on his or her experiences in order to achieve the stated goals for a four stage multi echelon SCN design.

### 4.1. Limitations and Findings

Other major techniques that can be considered prevalent in the literature include: GAs, a type of search technique that mimics natural selection and is capable of tackling various categories of combinatorial decision problems; data mining, which can be employed to provide insights and make decisions from large data sets; CBR, a cognitive psychological-based technique that solves new problems by retrieving gathered and saved cases of analogous problem-solving episodes and adapting them to the new problem at hand; and CBR is a technique that can be considered Other forms of artificial intelligence that are used in studies of SCM include simulated annealing, automated planning, association rules, tree-based models, hill climbing, k-means clustering, expert systems, heuristics, robot programming, stochastic simulation, Bayesian networks, the Physarum model, RBR, decision trees, and Gaussian models. These forms of AI are used less frequently than others. Studies on SCM have made use of these approaches, but not as often as studies have made use of ANNs, FL, ABSs, GA, data mining, CBR, swarm intelligence, or SVMs. This creates an intriguing gap that need to be addressed in further study and is something that has been done. In addition, our findings indicate that a number of AI techniques, such as NLP (machine–human interactions), TS (optimization, robot dynamics, and programming that focuses on creating intelligent robots), and MDP, require additional research and the adoption of these techniques in the industrial sector (a framework for modelling the decision-making process) [21–25].

## 5. Conclusion

It has been proven in this suggested work that a variety of unique concepts, approaches, and algorithms may be utilised to the design of integrated supply chain network architecture in order to optimise a structured supply chain network. On the other side, the six recognised organisational performance criteria are stakeholder satisfaction, innovation and learning, market performance, customer satisfaction, and financial success. As a consequence of this, the total performance metrics of the job that was presented are 94.12 percent, and the rates of accuracy, specificity, and sensitivity were discovered to be 94.12 percent, 92.15 percent, and 89.14 percent accordingly.

In addition, we discovered that the network-based structure of SCM and logistics gives a natural framework in which to deploy AI. This was discovered via our research. For example, a network of suppliers results in the production of significant quantities of data and calls for swift decision-making. As a result of this, using AI technologies for the study of large data and DSSs is highly suggested. In addition, supply chain management organisations are reliant on both physical and digital networks, both of which need to operate in harmony in order to be successful in the face of high volumes, lean asset allocation, poor margins, and stringent deadlines. AI makes it possible to optimise and improve network orchestration in a way that is both efficient and effective, both of which are impossible for humans to do. Therefore, research on interactive decision-making systems encourages a greater knowledge of AI solutions, and as a result, such study increases the capabilities of AI solutions. The utilisation of such systems makes it possible for AI to assist in the industry in question in redefining the practises that are currently in use by shifting operations from being reactive to being proactive, processes from being manual to being autonomous, services from being standardised to being personalised, and production planning from being predictive to being forecasting. The broad use of artificial intelligence is contingent on the development of more advanced computer chip technology. Because transportation is at the heart of logistics, the use of computer chips as a tracking mechanism is an absolutely necessary step. Research on such processes for the result of these technologies is required since tracking creates vast volumes of data that may be analysed and interpreted for a wide variety of applications. Automation of consumer interactions is a relatively new but potentially fruitful field that plays a major role in marketing. Voice or chatbots are examples of the next generation of customer care, which boasts excellent levels of efficiency and satisfactory returns on investment. The employment of these virtual assistants, which are designed to enable more in-depth conversations to take place between businesses and their clients, may prove to be very useful in the automation of customer support inquiries [26].

## Figures and Tables

**Figure 1:** Proposed network architecture.

**Figure 2:** Performance metrics.

**Figure 3:** MSE in presence of classifier.

**Figure 4:** MSE in presence of non-gaussian noise.

**Table 1:** Performance metrics of the proposed work.

S. No	Weights for objectives		Best fitness 1	Best fitness 2	Overall objective	Objective 1	Objective 2
	*w*1	*w*2				TMC/TSCC	
1	0.1	0.9	0.896485	0.846702	0.85168	1344727	0.71123
2	0.2	0.8	0.941887	0.831171	0.853314	1412830	0.698184
3	0.3	0.7	0.889595	0.847573	0.860179	1334392	0.711961
4	0.4	0.6	0.870228	0.864839	0.866995	1305342	0.726465
5	0.5	0.5	0.874051	0.863394	0.868723	1311037	0.725251
6	0.6	0.4	0.800067	0.921406	0.848603	1200101	0.773981
7	0.7	0.3	0.831129	0.89469	0.850198	1246694	0.75154
8	0.8	0.2	0.815808	0.909032	0.834453	1223712	0.763587
9	0.9	0.1	0.784989	0.932937	0.799784	1177483	0.783667

## Data Availability

The data that support the findings of this study are available on request from the corresponding author.
